# Inhibitory Effect of Multimodal Nanoassemblies against Glycative and Oxidative Stress in Cancer and Glycation Animal Models

**DOI:** 10.1155/2021/8892156

**Published:** 2021-04-09

**Authors:** Hamda Khan, Mohd Waseem, Mohammad Faisal, Abdulrahman A. Alatar, Ahmed A. Qahtan, Saheem Ahmad

**Affiliations:** ^1^Laboratory of Glycation Biology and Metabolic Disorder, Integral Research Centre-1, Department of Biosciences, Integral University, Lucknow 226026, India; ^2^Department of Zoology, Jagdam College, Jai Prakash University, Chapra, Bihar, India; ^3^Department of Botany and Microbiology, College of Sciences, King Saud University, Riyadh, Saudi Arabia; ^4^Department of Clinical Laboratory Sciences, College of Applied Medical Sciences, University of Hail, Hail, Saudi Arabia

## Abstract

In recent years, there has been a progress in the study of glycation reaction which is one the possible reason for multiple metabolic disorders. Glycation is a nonenzymatic reaction between nucleic acids, lipids, and proteins resulting into the formation of early glycation products that may further lead to the accumulation of advanced glycation end products (AGEs). The precipitation of AGEs in various cells, tissues, and organs is one of the factors for the initiation and progression of various metabolic derangements including the cancer. The AGE interaction with its receptor “RAGE” activates the inflammatory pathway; yet, the downregulation of RAGE and its role in these pathways are not clear. We explore the effect of anticancer novel nanoassemblies on AGEs to determine its role in the regulation of the expression of RAGE, NFƙB, TNF-*α*, and IFN-*γ*. This paper is based on the in vivo and in vitro study in glycation and lung cancer model systems. Upon the treatment of nanoassemblies in both the model systems, we observed a protective effect of nanoassemblies over the inhibition of glycative and oxidative stress via mRNA expression analysis. The mRNA expression results corroborated with the reactive oxygen species (ROS), carboxy-methyl-lysine (CML), and fluorescence studies. In this study, we found that the presence of common factors for glycation and lung cancer is oxidative and glycative stress. This oxidation and glycation might be responsible for the initiation of inflammation which may further lead to uncontrolled growth of cells leading to cancer. This can be a strong association between lung cancer and glycation reaction. The intervention of the anticancer and antiglycation effects of multimodal nanoassemblies throughout the study promises a new pathway for cancer research.

## 1. Introduction

Glycation is the nonenzymatic reaction between free amino groups of proteins and nucleic acids and free carbonyl groups of reducing sugars which damage or alter the protein structure and functions [1–6]. The damage caused to biological macromolecules through glycation and its final product, advanced glycation end products (AGEs), is the focal point of this study which leads to multiple metabolic disorders. AGEs are responsible for many diseases like, diabetes, ageing, and neurological disorders. Previous studies have shown that AGEs are also responsible for lung, breast, prostate, liver and head and neck cancer [7–10]. Different AGEs such as carboxy-methyl-lysine (CML), pentosidine, and fructosamine behave differently in the initiation and progression of cancer [11–13]. Several drugs have been tested to serum proteins, and new antiglycation agents have been identified from a diverse class of chemicals [14]. The nanoparticle-based drug delivery systems have unique properties as compared with traditional drug formulations. Nowadays, these are being extensively used in the treatment of diseases, such as diabetes, cardiovascular diseases, and cancer [15, 16]. In the present study, we used multifunctional nanoassemblies using perfluoroaryl-labelled albumin (PFT-Hcy-HSA) with a fluorescent dye (Cy7) and anticancer mononucleotide (trifluorothymidine, TFT). The size and shape of the nanoassemblies were examined by transmission electron microscopy. Human serum albumin (HSA) was used as a drug delivery carrier to construct a drug, and an approachable model is necessary for targeting drug delivery in cancer therapy. Also, HSA is an attractive model used to design multifunctional nanoassemblies for the theranostic approach. It acts as a drug carrier for a long time either by direct genetic fusion or conjugation or by a noncovalent association of a drug with the protein. The synthesized nanoassemblies, viz., PFT-HSA-TFT-Cy7 and PFT-Hcy-HSA-Cy7, were gifted by our collaborators, Professor Tatyana S. Godovikova and Professor Vladimir Silnikov, from ICBFM, RAS, and Novosibirsk, Russia.

There is a gradual increase in lung cancer subjects in the past decade which prompt us to perform this study [17]. We choose to perform the antiglycation study by comparing it with the anticancer activity. This has been monitored in lung cancer and glycation animal model. In our prior experiments, we developed two in vivo models based on the glycation and lung cancer model and one in vitro model based on lung cancer A-549 cell line [18]. Previously, the anticancer study was done on lung cancer cell line A-549 and breast cancer cell line MCF–7 in the presence of PFT-Hcy-HSA-Cy7 [19]. The antiglycation effects were examined by measuring fluorescent and nonfluorescent AGEs, while the anticancer effects were examined by observing inhibition in tumor growth, H&E staining, cell proliferation, and intracellular reactive oxygen species (ROS). Besides, the receptor of advanced glycation end products (RAGE) and AGEs activates the inflammatory reactions involved in the generation and progression of cancer. The AGE-RAGE axis leads to the activation of transcription factors, cytokines, and other interleukins that modify the signaling pathways by inducing the oxidation and inflammation [20]. The AGE-RAGE interaction mediates cell stress and triggers the inflammatory pathways by activating the signal transduction pathway (Scheme 1). Hence, we aim to target the signaling pathways which are involved in the initiation of cancer such as NFƙB, TNF-*α*, and IFN-*γ*. We analyzed the gene expression of NFƙB, TNF-*α*, and IFN-*γ* in the presence or absence of PFT-HSA-TFT-Cy7 and PFT-Hcy-HSA-Cy7.

## 2. Materials and Methods

### 2.1. Materials

Sprague-Dawley rats, Swiss albino mice, newly synthesized nanoassemblies (PFT-HSA-TFT-Cy7 and PFT-Hcy-HSA-Cy7), CML detection ELISA kit (bioassay technology laboratory), TRIzol Reagent (Ambion), primers (Eurofins), Revert Aid First Strand cDNA Synthesis Kit (Thermo Scientific), real-time PCR (Himedia). Hi-SYBr Master Mix, Agarose, Tris buffer, ethidium bromide, bromophenol blue, Protein Estimation Kit (G Biosciences), DNPH, methylglyoxal, bovine serum albumin, PBS, antibiotic antimycotic solution, and trypsin (all these chemicals were purchased from Himedia), glucometer (One Touch Select simple), 0.2 *μ*m syringe filter (Sartorius), DCFDA dye, nitrosodiethylamine, alloxan monohydrate (all these chemicals were purchased from Sigma Aldrich), UV-spectrophotometer (Eppendorf), spectrofluorometer (Agilent technologies, Carry Eclipse), phenobarbitone (Abbot), RPMI (Cell Clone), fetal bovine serum (Gibco), and RNA later (Invitrogen).

### 2.2. Ethics Statement

The animals were treated with the utmost care, and treatments were done with minimum pain. The rats and mice (6 per cage) were housed and acclimatized to the animal house environment for 10 days at room temperature (25°C) with 12 hour light and dark cycles. The in vivo work was approved by the Institutional Animal Ethical Committee (IAEC) of Integral University, Lucknow, India (1213/GO/ac/2008/CPCSEA).

### 2.3. Experimental Procedure for the Treatment of Nanoassemblies in the Glycation Animal Model

Sprague-Dawley rats (200–250 g) were being injected with alloxan (100 mg/kg body) in a starved condition via intraperitoneal routes [18]. All the animal groups were kept on 10% glucose for the next 24 hours to prevent hypoglycemia. The treatment group was given with 5 *μ*M concentration of both the nanoassemblies that is PFT-HSA-TFT-Cy7 and PFT-Hcy-HSA-Cy7. Fasting blood glucose (FBG) was checked after 24 hours of each dosing of alloxan. The procedure for the development of the glycation animal model as well as its treatment procedure with or without the presence of nanoassemblies has been provided in Table 1. All the rats were anesthetized using diethyl ether and sacrificed. Blood was collected by heart puncture. A sample of the kidney tissue was preserved in RNA later.

### 2.4. Experimental Procedure for the Treatment of Nanoassemblies in the Lung Cancer Animal Model

The anticancer activity of the nanoassemblies in the lung cancer animal model has been done by the oral dosing of both nanoassemblies at 1 *μ*M and 3 *μ*M. We developed the lung cancer animal model in Swiss albino mice with NDEA and PB [18]. The experimental procedure of the development of lung cancer, as well as the inhibitory effect of nanoassemblies, has been briefly explained in Table 2. After 50 days, all the mice were anesthetized using diethyl ether and sacrificed. Blood was collected through heart puncture. The lung tissue was isolated and preserved in 10% formalin and RNA later separately. The fragments from the lung tumur tissues were embedded in paraffin blocks and sectioned at 3–5 *μ*m for histological analyses, and then each histological slide from each block was stained with hematoxylin (H) and eosin (E). Each experimental group was examined carefully using a light microscope with magnification at 40x.

### 2.5. Experimental Procedure for the Treatment of Nanoassemblies in the vitro Model System

The A-549 lung cancer cell line (5000 cells/well) in 100 *μ*l of complete medium was seeded in 96-well plates. After 4 hours of incubation allowing the cells to attach to the bottom of the well, the medium was renewed for a further 24 hours of incubation along with the addition of 25 mM of BSA-MG-AGEs (100 *μ*g) or unmodified BSA (100 *μ*g). The BSA-MG-AGEs were prepared by our previous method (18), and this is a glycation reaction of a protein bovine serum albumin (BSA) and methylglyoxal (MG). The wells were treated with different concentrations of PFT-HSA-TFT-Cy7 and PFT-Hcy-HSA-Cy7 at 1 *μ*M, 3 *μ*M, and 5 *μ*M, respectively. All the experiments were performed in duplicate. The cells were then lysed with 100 *μ*l/well of TRIzol Reagent. The cell lysates were collected in microcentrifuge tubes and stored at -20°C. For cell proliferation effects, 30,000 cells were seeded in the six-well plate containing 2 ml of media. After 4 hours of incubation allowing the cells to attach to the bottom of the well, the media was renewed for a further 24 hours of incubation along with the addition of 25 mM of BSA-MG-AGEs (100 *μ*g) or unmodified BSA (100 *μ*g) in the presence of PFT-HSA-TFT-Cy7 and PFT-Hcy-HSA-Cy7 at 1 *μ*M, 3 *μ*M, and 5 *μ*M, respectively. Cell counts were taken by using hemocytometer as previously suggested [21].

### 2.6. Estimation of Oxidative Stress with or without the Presence of PFT-HSA-TFT-Cy7 and PFT-Hcy-HSA-Cy7

The oxidative stress in the glycation, as well as the lung cancer animal model in the presence of nanoassemblies, has been detected through estimation of the carbonyl content and malondialdehyde (MDA) content. The carbonyl content was determined in the serum samples of the glycation animal model as well as the lung cancer animal model along with their treatment group, respectively, by using 2,4-dinitrophenylhydrazine (2,4 DNPH). The absorbance was read at 360 nm, and the carbonyl content was determined by using the extinction coefficient of 22,000 M^−1^ cm^−1^ [22]. Similarly, the thiobarbituric acid reactive substance (TBARS) assay is to perform for the detection of the MDA content, which is formed during the intermediate stage of the glycation reaction also. 100 *μ*l serum sample was diluted with 500 *μ*l of phosphate buffer saline (PBS). One ml TBA-TCA-HCl reagent was added to each diluted sera sample at room temperature. The pink supernatant was observed after boiling the reaction for 15 minutes at 100°C. The pink supernatant was read at 535 nm. The concentration was plotted by the obtained absorbance against the standard graph. The optical density of the pink color formed is directly proportional to the concentration of serum MDA in the given sample. The AGE-induced formation of intracellular ROS of the in vitro model was measured by using dichlorodihydrofluorescein diacetate (H2DCFDA) as described previously with slight modification [23]. A549 cells were seeded in 96-well plates (3000 cell/well) and incubated at 37°C with 5% CO2 for about 24 h. The cells were treated with 100 *μ*g/ml of 25 mM bovine serum albumin AGE (BSA-AGEs) samples for 24 h in the presence of both the nanoassemblies at 1 *μ*M, 3 *μ*M, and 5 *μ*M, respectively. After incubation, DCFDA was added (10 *μ*M), and the plate was incubated for 30 min in dark. DCFDA was removed, and wells were washed once with PBS and finally, cells were suspended in 100 *μ*l of PBS. The plate was read at 485/528 (excitation/emission) at 100% sensitivity, and readings were presented as relative fluorescence unit for ROS generation. The cells without treatment were considered as control.

### 2.7. Estimation of Glycative Stress with or without the Presence of PFT-HSA-TFT-Cy7 and PFT-Hcy-HSA-Cy7

The estimation of glycative stress was done through the detection of fluorescent and nonfluorescent AGEs. The fluorescent intensity (F.I.) of the serum samples (diluted to 1 : 50) and cell lysates was measured at 370 nm excitation/440 nm emissions, 360 nm excitation/460 nm emissions, and 420 nm excitation/440 nm emission of the lung cancer animal model, glycation animal model, and in vitro model system, respectively [18]. The % increase of fluorescent intensity (F.I.) of the treated, as well as nontreated samples, was calculated by the following given method:

%increase of F.I = (F.I.of test − F.I.of control)/(F.I.of test) × 100.

For CML detection, we used the commercially available ELISA kit for all the three model systems with or without the presence of nanoassemblies. The treated and nontreated serum samples and cell lysates were added in the wells after dilution with PBS in the ratio of 1 : 100. After incubation, the kit protocol has been followed until the end of the reaction. The reaction was stopped by the addition of an acidic stop solution, and absorbance is measured at 450 nm.

### 2.8. RNA Isolation and Quantification

Total number of RNA was extracted from the tissue of the lung cancer and glycation model system. The isolation was done by using the TRIzol Reagent method. The minced tissue sample and cell lysates were centrifuged at 14,000 rpm for 10 minutes at 4°C. Transfer the supernatant in a new tube containing chloroform in the ratio of 1 : 3. Keep the sample at room temperature after shaking vigorously for 30 seconds. Repeat the centrifugation process once again. Now, carefully transfer the supernatant in a fresh tube containing ice chilled isopropanol. Incubate the mixture for 15 minutes at room temperature. Again, repeat the centrifugation process. Wash the RNA pellet with 80% ethanol. Use DEPC treated water to dissolve the RNA pellet finally. The concentration of isolated RNA from tissues samples and cell lysates was quantified by Nanodrop. Blank was set through a solvent (DEPC treated water) used to dissolve RNA. RNA sample was mixed by gentle vortexing and inversion and placed 1 *μ*l RNA solution on instrument plate for concentration measurement. The ratio of A260/A280 is used as a relative measure of the nucleic acid/protein content of an RNA sample. The typical A260/A280 for isolated RNA is 2.0, and a lesser ratio (2.0 < 1.8) indicates DNA contamination. Agarose gel electrophoresis was performed to check the quality of RNA on 1.3% by using 1× TBE buffer.

### 2.9. cDNA Synthesis

cDNA synthesis was done as per the manufacturer's (Thermo scientific) protocol. Thermo scientific c-DNA synthesis kit is a complete system for efficient synthesis of first-strand cDNA. The final volume was 20 *μ*l. The procedure for cDNA synthesis from a kit is as given below in Table 3.

Add the following reagent on ice in a sterile condition after thawing properly. Mix gently and spin it for proper mixing. The reaction is extended at its first stage for 62 minutes at 42°C. At the second stage, the reaction is heated at 70°C for 5 minutes to inactivate the enzyme.

### 2.10. Sequences of Chosen Primer

The primers used in the mRNA expression study are shown in Table 4. The desired primer sequences were designed through Primer 3.0 software.

### 2.11. Real-Time PCR

The real-time PCR analysis of the tissue samples and cell lysates was assisted after the isolation and quantification of RNA followed by the synthesis of cDNA. The reaction volume is 13 *μ*l per reaction following the RT-PCR standard condition, i.e., 95°C for 5 min at hold stage, 95°C for 30 sec, 59°C for 30 sec, and 72°C for 35 sec×40 cycles at PCR stage, and 95°C for 20°sec, 60°C for 60°sec, and 95°C for 30 sec at melting stage. The cycle of the threshold (Ct) value of each sample was calculated by using the Livak method for the fold change expression, i.e., 2^**-*ΔΔ*Ct**^.

### 2.12. Statistical Analysis

Data are presented as mean ± SD, and statistical significance of the data was determined by Microsoft Excel (version 2010). One-way ANOVA was performed by Graph Pad Prism 8. A value of *P* ≤ 0.05 was considered statistically significant.

## 3. Results

### 3.1. Lowering of Blood Glucose by PFT-HSA-TFT-Cy7 and PFT-Hcy-HSA-Cy7

The level of FBG was measured as a strong factor in the glycation animal model. The % decrease in the FBG has been observed as 4.6%, 15.73%, 31.60%, and 61.74% (group 3) respective to the control group with the treatment of PFT-HSA-TFT-Cy7 at week 1^st^, week 2^nd^, week 3^rd^, and week 4^th^. The % decrease in the level of FBG in the presence of PFT-Hcy-HSA-Cy7 has been calculated as 4.06%, 10.11%, 31.32%, and 57.48% (group 4) respective to the control group at 1^st^ week, 2^nd^ week, 3^rd^ week, and 4^th^ week (Figure 1(a)).

### 3.2. Inhibition of Tumor Growth in the Presence of PFT-HSA-TFT-Cy7 and PFT-Hcy-HSA-Cy7

Hematoxylin and Eosin (HE) staining showed a specific histological change in the pattern of histological sections under the treatment of PFT-HSA-TFT-Cy7 and PFT-Hcy-HSA-Cy7 (Figure 1(c)). Tumor growth was characterized by a tumor node which that was almost negligible in the treatment groups. A marked reduction in tumor node was seen in Figure 1(b).

### 3.3. Inhibitory Effect of PFT-HSA-TFT-Cy7 and PFT-Hcy-HSA-Cy7 against Oxidative Stress in Glycation Animal Model and Lung Cancer Animal Model

In the lung cancer animal model, we observed 26.88% and 33.76% decrease in the level of the carbonyl content with the treatment of PFT-HSA-TFT-Cy7 at 1 *μ*M and 3 *μ*M while 31.55% and 44.54% decrease in the carbonyl content in the presence of PFT-Hcy-HSA-Cy7 at 1 *μ*M and 3 *μ*M. On the other hand, in the glycation animal model, we observed 39.14% and 42.90% inhibition of the carbonyl content with the treatment of PFT-HSA-TFT-Cy7 and PFT-Hcy-HSA-Cy7 at 5 *μ*M (Figure 2(a)). Similarly, the decrease in the MDA level in lung cancer animal model was observed as 21.78% and 43.01% in the presence of PFT-HSA-TFT-Cy7 at 1 *μ*M and 3 *μ*M and 11.73% and 35.75% in the presence of PFT-Hcy-HSA-Cy7 at 1 *μ*M and 3 *μ*M respective to their control. The glycation animal model showed 45.97% and 28.16% inhibition of the MDA content with the treatment of both the nanoassemblies that is PFT-HSA-TFT-Cy7 and PFT-Hcy-HSA-Cy7 at 5 *μ*M (Figure 2(b)).

### 3.4. Inhibition in Cell Proliferation and Intracellular ROS of A-549 Cell Line by PFT-HSA-TFT-Cy7 and PFT- Hcy-HSA-Cy7

The cell counting via hemocytometer of each treated wells showed cell proliferation between control, native BSA, and 25 mM MG modified BSA in the presence of PFT-HSA-TFT-Cy7 and PFT-Hcy-HSA-Cy7. The result we obtained indicates that there is a decrease in cell proliferation at1*μ*M, 3 *μ*M, and 5 *μ*M of PFT-HSA-TFT-Cy7 and PFT-Hcy-HSA-Cy7. A maximum of 33.24% and 25.39% inhibition in cell growth was observed at a maximum concentration of PFT-HSA-TFT-Cy7 and PFT-Hcy-HSA-Cy7, respectively, as compared to their control (Figure 3(a)). The in vitro work investigation indicates a significant decrease in ROS with the treatment of PFT-HSA-TFT-Cy7 and PFT-Hcy-HSA-Cy7. PFT-HSA-TFT-Cy7 inhibits 25.11%, 29.49%, and 39.56% level of ROS while PFT-Hcy-HSA-Cy7 inhibits 25.80%, 37.05%, and 50.09% at 1 *μ*M, 3 *μ*M, and 5 *μ*M, respectively as compared to their respective control (Figure 3, Table 5).

### 3.5. Inhibition of Glycative Stress in the Presence of PFT-HSA-TFT-Cy7 and PFT-Hcy-HSA-Cy7

Moreover, inhibition of glycative stress is measured by inhibition in fluorescent AGEs and nonfluorescent AGEs. The lowering of fluorescent AGEs in the glycation animal model has been calculated as 20.23% and 26.33% with the treatment of PFT-HSA-TFT-Cy7 and PFT-Hcy-HSA-Cy7 at 5 *μ*M (Figure 4(b)). The lung cancer animal model shows 8.7% and 21.05% reduction in fluorescent AGEs during the treatment with PFT-HSA-TFT-Cy7 at 1 *μ*M and 3 *μ*M; on the other hand, the PFT-Hcy-HSA-Cy7 shows 6.57% and 19.29% inhibition in fluorescent AGEs at 1 *μ*M and 3 *μ*M, respectively (Figure 4(a)). Furthermore, our in vitro model shows 7.09%, 14.42%, and 26.65% inhibition in the presence of PFT-HSA-TFT-Cy7 at 1 *μ*M, 3 *μ*M, and 5 *μ*M, respectively (Figure 4(c)). PFT-Hcy-HSA-Cy7 shows 2.2%, 26.66%, and 31.54% inhibition as compared to their respective controls at 1 *μ*M, 3 *μ*M, and 5 *μ*M, respectively (Figure 4(d)).

The nonfluorescent AGEs, i.e., CML, have been largely known AGEs found in food. Previously, we observed that MG which is a potent precursor of AGEs can be able to further generate CML in glycation and lung cancer animal model [16]. This observation encourages us to go through the inhibitory activity of the provided nanoassemblies against CML. We found % decrease in the CML content as 33.33% and 35.00% with the treatment of PFT-HSA-TFT-Cy7 and PFT-Hcy-HSA-Cy7 at 5 *μ*M in the glycation animal model (Figure 5(b)). The lung cancer animal model showed 23.18% and 28.2% decrease in the CML content at 1 *μ*M and 3 *μ*M, respectively, in the presence of PFT-HSA-TFT-Cy7. Similarly, in the same model, we observed 23.01% and 27.33% inhibitory activity in the presence of PFT-Hcy-HSA-Cy7 at 1 *μ*M and 3 *μ*M, respectively (Figure 5(a)). After the successful in vivo inhibition of CML, we further escalated our study to in vitro CML content inhibition. The maximum inhibition in the CML content was recorded as 38.7% and 33.77% with the treatment of PFT-HSA-TFT-Cy7 and PFT-Hcy-HSA-Cy7 as compared to their respective control (Figure 5(c)).

### 3.6. RAGE Expression in All the Three Samples with or without the Presence of PFT-HSA-TFT-Cy7 or PFT-Hcy-HSA-Cy7

The RAGE mRNA levels were increased in the tissue sample of the glycation animal model as compared to its control group, with an average increase of 3.0-fold (*P* < 0.008) (Figure 6(b)), while the RAGE mRNA levels of the tissue sample of the cancer animal model were increased as compared to its control group with an average increase of 2.9-fold (*P* < 0.001) (Figure 6(a)). The RAGE expression was significantly upregulated in the BSA-MG-AGEs/A549 lung cancer cell line as compared to the control group, with an average increase of 9.7-fold (*P* < 0.001) (Figure 6(c)). Similarly, the treatment group of the glycation model system in the presence of PFT-HSA-TFT-Cy7 and PFT-Hcy-HSA-Cy7 shows significantly downregulated level of RAGE mRNA, with an average decrease in fold change as 2.3-fold and 2.0-fold at 5 *μ*M of concentration, respectively (Figure 6(b)). While on the other hand, the treatment group of the cancer tissue with PFT-HSA-TFT-Cy7 and PFT-Hcy-HSA-Cy7 shows a significant decrease in the level of RAGE mRNA, with an average decrease in fold change as 2.0-fold and 1.91-fold at 1 *μ*M and 2.5-fold and 1.6-fold at 3 *μ*M concentration of nanoassemblies (Figure 6(a)). The treatment group of the in vitro model system also showed downregulation, and the fold change in the presence of PFT-HSA-TFT-Cy7 has been noted as 7.9-fold, 6.85-fold, and 3.5-fold as compared to their respective control at 1 *μ*M, 3 *μ*M and 5 *μ*M, respectively. While in the presence of PFT-HSA-TFT-Cy7, it showed 7.1-fold, 5.05-fold, and 3.4-fold change at 1 *μ*M, 3 *μ*M, and 5 *μ*M, respectively (Figure 6(c)).

### 3.7. TNF-*α* Expression in All the Three Samples with or without the Presence of PFT-HSA-TFT-Cy7 or PFT-Hcy-HSA-Cy7

The TNF-*α* mRNA levels were increased in the tissue sample of the glycation animal model as compared to its control group, with an average increase of 2.04-fold (*P* < 0.005) (Figure 6(b)), while the TNF-*α* mRNA levels of the tissue sample of the cancer animal model were increased as compared to its control group with an average increase of 2.9-fold (*P* < 0.005) (Figure 6(a)). The TNF-*α* expression was significantly upregulated in the BSA-MG-AGEs/A549 lung cancer cell line as compared to the control group, with an average increase of 7.49-fold (Figure 6(e)). The treatment group of the glycation model system in the presence of PFT-HSA-TFT-Cy7 and PFT-Hcy-HSA-Cy7 shows significantly downregulated level of TNF-*α* mRNA, with an average decrease in fold change as 1.1-fold and 1.4-fold at 5 *μ*M of concentration, respectively (Figure 6(b)). While on the other hand, the treatment group of the cancer tissue with PFT-HSA-TFT-Cy7 and PFT-Hcy-HSA-Cy7 shows a significant decrease in level of TNF-*α* mRNA, with an average decrease in fold change as 1.9-fold and 2.3-fold at 1 *μ*M and 1.5-fold and 1.9-fold at 3 *μ*M with respect to their controls (Figure 6(a)). The treatment group of the in vitro model system shows 5.8-fold, 5.1-fold, and 3.6-fold change in the presence of PFT-HSA-TFT-Cy7 at 1 *μ*M, 3 *μ*M, and 5 *μ*M, respectively. Similarly, the treatment group of the in vitro model system in the presence of PFT-Hcy-HSA-Cy7 showed 6.6-fold, 5.6-fold, and 2.7-fold change in the presence of 1 *μ*M, 3 *μ*M, and 5 *μ*M, respectively (Figure 6(e)).

### 3.8. NF*κ*B Expression in All the Three Samples with or without the Presence of PFT-HSA-TFT-Cy7 or PFT-Hcy-HSA-Cy7

The NF*κ*B mRNA levels were increased in the tissue sample of the glycation animal model as compared to its control group, with an average increase of 3.9-fold (Figure 6(b)), while the NF*κ*B mRNA levels of the tissue sample of the cancer animal model were increased as compared to its control group with an average increase of 4.1-fold (*P* < 0.001) (Figure 6(a)). The NF*κ*B expression was significantly upregulated in the BSA-MG-AGEs/A549 lung cancer cell line as compared to the control group, with an average increase of 10.1-fold (Figure 6(d)). The treatment group of the glycation animal model and cancer animal model in the presence of PFT-HSA-TFT-Cy7 and PFT-Hcy-HSA-Cy7 showed downregulation (Figures 6(a) and 6(b)). PFT-HSA-TFT-Cy7 and PFT-Hcy-HSA-Cy7 showed 2.8-fold and 1.9-fold at 5 *μ*M of concentration, in the glycation animal model (Figure 6(b)), while the treatment group of the cancer tissue with PFT-HSA-TFT-Cy7 and PFT-Hcy-HSA-Cy7 showed a decrease in the level of NF*κ*B mRNA, with an average decrease in fold change as 2.2-fold and 2.7-fold at 1 *μ*M and 1.6-fold and 1.5-fold at 3 *μ*M concentration of nanoassemblies (Figure 6(a)). The treatment group of the in vitro model system showed fold change as 7.9-fold, 5.4-fold, and 4.1-fold in the presence of PFT-HSA-TFT-Cy7 at 1 *μ*M, 3 *μ*M, and 5 *μ*M, respectively, as compared to their respective control, while the same group in the influence of PFT-Hcy-HSA-Cy7 showed the fold change as 5.5-fold, 4.9-fold, and 4.1-fold at 1 *μ*M, 3 *μ*M, and 5 *μ*M, respectively (Figure 6(d)).

### 3.9. IFN-*γ* Expression in All the Three Samples with or without the Presence of PFT-HSA-TFT-Cy7 or PFT-Hcy-HSA-Cy7

The IFN-*γ* mRNA levels were increased in the tissue sample of the glycation animal model as compared to its control group, with an average increase of 1.9-fold (*P* < 0.005) (Figure 6(b)), while the IFN-*γ* mRNA levels of the tissue sample of the cancer animal model were increased as compared to its control group with an average increase of 5.7-fold (*P* < 0.005) (Figure 6(a)). Similarly, the IFN-*γ* expression was significantly upregulated in the BSA-MG-AGEs/A549 lung cancer cell line as compared to the control group, with an average increase of 9.7-fold (Figure 6(f)). The treatment group of the glycation animal model in mediation of PFT-HSA-TFT-Cy7 showed downregulation. PFT-HSA-TFT-Cy7 and PFT-Hcy-HSA-Cy7 show significantly downregulated level of IFN-*γ* mRNA, with an average decrease in fold change as 1.59-fold and 1.3-fold at 5 *μ*M of concentration (Figure 6(b)). While on the other hand, the treatment group of the cancer tissue with PFT-HSA-TFT-Cy7 and PFT-Hcy-HSA-Cy7 shows a significant decrease in level of IFN-*γ* mRNA, with an average decrease in fold change as 3.3-fold and 3.2-fold at 1 *μ*M and 3.0-fold and 1.7-fold at 3 *μ*M concentration of nanoassemblies (Figure 6(a)). The treatment group of the in vitro model system shows 6.6-fold, 5.5-fold, and 2.8-fold change in the presence of PFT-HSA-TFT-Cy7 at 1 *μ*M, 3 *μ*M, and 5 *μ*M, respectively, with respect to their control (Figure 6(f)). Similarly, the treatment group of the in vitro model system in the presence of PFT-Hcy-HSA-Cy7 showed 5.9-fold, 3.6-fold, and 2.9 fold at 1 *μ*M, 3 *μ*M, and 5 *μ*M, respectively, as compared to their control (Figure 6(f)).

## 4. Discussion

Cancer is a leading health problem globally with around 14 million new cases recorded each year [24]. Hyperglycemia, energy imbalance, chronic inflammation, and insulin resistance are underlying mechanisms of cancer development. Moreover, AGEs are also involved in cancer progression. AGEs regulate cancer progression by activating its receptor RAGE. In our previous study, we established a link between glycation and lung cancer animal model [24]. While in this study, we used new multimodal nanoassemblies which are anticancerous in nature and designed as fluorinated nucleotide conjugated with dually labeled albumin. The report on its anticancer activity has been previously published [25], while in the current research, we are trying to find out its antiglycation property since we believe that AGE reduction might combat the cancer risk as well. Cancer is uncontrollable while AGEs are not; therefore, it is better to control cell growth by choosing an alternate pathway which might be an intermediate link for cancer growth. AGEs are supposed to be one of them [18, 26]. We evaluated the inhibitory effect of PFT-HSA-TFT-Cy7 and PFT-Hcy-HSA-Cy7 on glucose in our glycation animal model. The maximum inhibition in the FBG level was observed on the fourth week which was recorded to be 61.7% by PFT-HSA-TFT-Cy7 (5 *μ*M) and 57.65% by PFT-Hcy-HSA-Cy7 (5 *μ*M) (Figure 1(a)). Furthermore, we identified its effect against glycative stress by measuring nonfluorescent AGEs “CML” and fluorescent AGEs. The inhibition of CML in the glycation animal model was 33.33% in the presence of PFT-HSA-TFT-Cy7 at 5 *μ*M concentration. Meanwhile, the inhibition via PFT-Hcy-HSA-Cy7 was recorded to be 35% against CML at the same concentration (Figure 5(b)). PFT-HSA-TFT-Cy7 and PFT-Hcy-HSA-Cy7 also showed an inhibitory effect against fluorescent AGEs. We observed 20.23% and 26.33% inhibition of the fluorescent AGEs by PFT-HSA-TFT-Cy7 and PFT-Hcy-HSA-Cy7, respectively (Figure 4(b)). Our result shows that the PFT-HSA-TFT-Cy7 and PFT-Hcy-HSA-Cy7 demonstrated effective inhibition of the fluorescent and nonfluorescent AGEs. Similarly, we observed inhibition in the growth of tumor node in our in vivo cancer animal model (Figure 1(b)). Moreover, the presence of fluorescent and no-fluorescent AGEs in the cancer animal model was also inhibited in the presence of these nanoassemblies (Figures 4(a) and 5(a)). PFT-HSA-TFT-Cy7 lowered the CML content by 23.18% and 28.2% at 1 *μ*M and 3 *μ*M, respectively. Similarly, PFT-Hcy-HSA-Cy7 lowered the CML content by 23.01% and 27.33% at 1 *μ*M and 3 *μ*M, respectively. Additionally, PFT-HSA-TFT-Cy7 reduced the fluorescent AGEs in the lung cancer animal model by 8.7% and 21.05% at 1 *μ*M and 3 *μ*M, respectively, while PFT-Hcy-HSA-Cy7 showed 6.57% and 19.29% inhibition of fluorescent AGEs in the same model. We also noted a inhibition of the carbonyl content by 26.88% and 33.76% in the presence of PFT-HSA-TFT-Cy7, while 31.55% and 44.54% in the presence of PFT-Hcy-HSA-Cy7, both in the cancer animal model with respect to their control (Figure 2(a)). On the other hand, in the glycation animal model, we observed 39.14% and 42.90% inhibition of oxidative stress with the treatment of both nanoassemblies that is PFT-HSA-TFT-Cy7 and PFT-Hcy-HSA-Cy7 at 5 *μ*M, respectively (Figure 2(a)). The decrease in the MDA content was found to be 21.87% and 43.01% with the treatment from PFT-HSA-TFT-Cy7 at 1 *μ*M and 3 *μ*M, respectively, while 11.73% and 35.75% from PFT-Hcy-HSA-Cy7 at similar concentrations in the cancer animal model. On the other hand, in the glycation animal model, we noted 28.16% and 45.97% inhibition of the MDA content with the treatment of both nanoassemblies that is PFT-HSA-TFT-Cy7 and PFT-Hcy-HSA-Cy7 at 5 *μ*M, respectively (Figure 2(b)). Also, our in vitro experiments using A549 lung cancer cell line showed successful inhibition of glycative and oxidative stress under the influence of PFT-HSA-TFT-Cy7 and PFT-Hcy-HSA-Cy7. We observed a successful inhibition of ROS production compared to control. The sample treated with PFT-HSA-TFT-Cy at 5 *μ*M showed 39.56% maximum inhibition in the ROS level compared to BSA-MG-AGEs. On the other hand, the sample treated with PFT-Hcy-HSA-Cy7 at 5 *μ*M showed 50.09% maximum inhibition in ROS level compared to BSA-MG-AGEs (Figure 3(b)). In addition, we observed 26.65% and 31.54% maximum inhibition of fluorescent AGEs in the cell lysates with PFT-HSA-TFT-Cy and PFT-Hcy-HSA-Cy7, respectively, at 5 *μ*M concentration (Figures 4(c) and 4(d)).

RAGE alters cell signaling pathways and contributes to endothelial dysfunction via tumor necrosis factor-*α* (TNF-*α*). The interaction of AGEs with RAGE sets off a cascade of events leading to the modulation of the gene expression and loss of vascular and tissue homeostasis, the processes that contribute to cardiovascular diseases [26] lung cancer [27], pancreatic cancer [28], hepatocellular carcinoma [29], and various other forms of cancer as well [30, 31]. Hence, our study further analyzed the gene expression in both glycation and cancer tissues in the presence or absence of PFT-HSA-TFT-Cy7 and PFT-Hcy-HSA-Cy7. Our gene expression analysis revealed an increase in mRNA levels of RAGE, NFƙb, TNF-*α*, and IFN-*γ*. However, tissue samples in the presence of PFT-HSA-TFT-Cy7 and PFT-Hcy-HSA-Cy7 showed lowered expression of RAGE, NFƙb, TNF-*α*, and IFN-*γ*. Similarly, higher expression levels of RAGE, NFƙb, TNF-*α*, and IFN-*γ* were observed in the untreated sample in our in vitro model. Meanwhile, the samples with PFT-HSA-TFT-Cy7 and PFT-Hcy-HSA-Cy7 showed maximum downregulation of RAGE, NFƙb, TNF-*α*, and IFN-*γ* at the maximum concentration of nanoassemblies (5 *μ*M).

Since AGEs are implicated in type 2 diabetes mellitus as reported by us and others [32, 33], there is a strong link between diabetes and cancer [34]. Diabetes is associated with increased risk for some cancers like the liver, pancreas, endometrium, colon, breast, and bladder. The association between diabetes and some cancers may partly be due to shared risk factors between the two diseases, such as AGEs, aging, obesity, diet, and physical inactivity. Possible mechanisms for a direct link between diabetes and cancer include hyperinsulinemia, hyperglycemia, and inflammation [34]. This is the preliminary study in which we have seen the expression study at mRNA level only, and some glycation, oxidation, and inflammatory markers were only studied. This study further warrants to study the expression of the pathways at protein levels too by western blotting experiments.

## 5. Conclusion

Our findings from this study indicate that the nanoassemblies may play a protective role in cancer by inhibiting glycative and oxidative stress. This study is the first attempt to evaluate the antiglycation and anticancer activity simultaneously in the presence of newly synthesized nanoassemblies, i.e., PFT-HSA-TFT-Cy7 and PFT-Hcy-HSA-Cy7. In conclusion, our study suggests that preventing the formation of AGEs inside the body might lower the risk of cancer growth.

## Figures and Tables

**Scheme 1:** Schematic representation of AGE-RAGE axis activation leads to the increase in ROS and inflammatory markers like, TNF-*α* and NF*κΒ*. These are involved in the cell signaling pathways which are responsible for cancer initiation and progression.

**Figure 1:** (a) Lowering of blood glucose in the presence of PFT-HSA-TFT-Cy7 (group 3) and PFT-Hcy-HSA-Cy7 (group 4) in the glycation animal model. *P* value is <0.05. (b) Inhibition in tumor node in the presence of PFT-HSA-TFT-Cy7 and PFT-Hcy-HSA-Cy7 in the lung cancer animal model of the control group (A), cancer group (B), treatment group with PFT-HSA-TFT-Cy7 (D), and treatment group with PFT-Hcy-HSA-Cy7 (D). (c) Histological analysis of lung tissue section of the cancer animal model of a control group (E), cancer group (F), treatment group with PFT-HSA-TFT-Cy7 (G), and treatment group with PFT-Hcy-HSA-Cy7 (H).

**Figure 2:** (a) Lowering of the carbonyl content level in the presence of PFT-HSA-TFT-Cy7 and PFT-Hcy-HSA-Cy7 in the lung cancer and glycation animal model. (b) Lowering of MDA content level in the presence of PFT-HSA-TFT-Cy7 and PFT-Hcy-HSA-Cy7 in the lung cancer and glycation animal model. *P* value is <0.05.

**Figure 3:** (a) Lowering of cell proliferation in the presence of PFT-HSA-TFT-Cy7 and PFT-Hcy-HSA-Cy7. (b) Lowering of ROS in the presence of PFT-HSA-TFT-Cy7 and PFT-Hcy- HSA-Cy7. *P* value is <0.05.

**Figure 4:** (a) Spectrofluorometric emission spectra of the glycation animal model in the presence of PFT-HSA-TFT-Cy7 and PFT-Hcy-HSA-Cy7. (b) Spectrofluorometric emission spectra of the lung cancer animal model in the presence of PFT-HSA-TFT-Cy7 and PFT-Hcy-HSA-Cy7. (c) Spectrofluorometric emission spectra of the in vitro model system in the presence of PFT-HSA-TFT-Cy and (d) PFT-Hcy-HSA-Cy7.

**Figure 5:** (a) Lowering of the CML content in the presence of PFT-HSA-TFT-Cy7 and PFT-Hcy-HSA-Cy7 in the lung cancer animal model. (b) Lowering of the CML content in the presence of PFT-HSA-TFT-Cy7 and PFT-Hcy-HSA-Cy7 in the glycation animal model. (c) Lowering of the CML content in the presence of PFT-HSA-TFT-Cy7 and PFT-Hcy-HSA-Cy7 and in the in vitro model system.

**Figure 6:** Downregulation of RAGE, NF*κ*B, TNF-*α* and IFN-*γ* in the presence of PFT-HSA- TFT-Cy7 and PFT-Hcy-HSA-Cy7 in (a) the lung cancer animal model (*P* value is ^∗∗∗^ < 0.001, ^∗∗^ < 0.002, ^∗^ < 0.02), (b) glycation animal model (*P* value is ^∗∗∗^ < 0.001, ^∗∗^ < 0.002, ^∗^ < 0.02), and (c) in vitro model system (*P* value is ^∗∗∗^ < 0.001, ^∗∗^ < 0.002, ^∗^ < 0.02).

**Table 1:** Stepwise method for the inhibitory effect of nanoassemblies in the glycation animal model.

Step	Experiment (dosing) (30 days)	Group 1 (*n* = 6)	Group 2 (*n* = 6)	Group 3 (*n* = 6)	Group 4 (*n* = 6)
Step 1 (acclimatization for one week)	Diet and normal water	Pellet diet/water	Pellet diet/water	Pellet diet/water	Pellet diet/water

Step 2 (after overnight fasting)	^∗^FBG	Check FBG after overnight fasting	Check FBG after overnight fasting	Check FBG after overnight fasting	Check FBG after overnight fasting

Step 3	Alloxan induction/booster dose after one week (if required)	No induction	100 mg/kg alloxan induction	100 mg/kg alloxan induction	100 mg/kg alloxan induction

Step 4	Nanoassembly treatment after one dosing of alloxan	No treatment	No treatment	5 *μ*M of PFT-HSA-TFT-Cy7	5 *μ*M of PFT-Hcy-HSA-Cy7

Step 5	Glucose	Normal water	10% glucose in drinking water daily for 30 days	10%glucose in drinking water daily for 30 days	10% glucose in drinking water daily for 30 days

^∗^FBG: fasting blood glucose.

**Table 2:** Stepwise method for the inhibitory effect of nanoassemblies in the lung cancer animal model.

Step	Experiment (dosing) (50 days)	Group 1 (*n* = 6)	Group 2 (*n* = 6)	Group 3 (*n* = 6)	Group 4 (*n* = 6)
Step 1 (acclimatization for one week)	Diet and normal water	Pellet diet/water	Pellet diet/water	Pellet diet/water	Pellet diet/water

Step 2	NDEA	No NDEA	100 ppm of NDEA in drinking water for initial 15 days	100 ppm of NDEA in drinking water for initial 15 days	100 ppm of NDEA in drinking water for initial 15 days

Step 3	500 ppm of PB	No PB	100 ppm of NDEA in drinking water along with 500 ppm PB for remaining 35 days	100 ppm of NDEA in drinking water along with 500 ppm PB for remaining 35 days	100 ppm of NDEA in drinking water along with 500 ppm PB for remaining 35 days

Step 4	Nanoassembly treatment	No treatment	No treatment	1 *μ*M (3mice) and 3 *μ*M (3 mice) of PFT-HSA-TFT-Cy7	1 *μ*M (3 mice) and 3 *μ*M (3 mice) of PFT-Hcy-HSA-Cy7

**Table 3:** Protocol of cDNA synthesis.

Reagents and samples	Volume
Control GAPDH RNA (50 ng/*μ*l)	2 *μ*l
Oligo (dT)18 primer or random hexamer primer or reverse GAPDH primer	1 *μ*l
5× reaction buffer	4 *μ*l
RiboLock RNase inhibitor (20 U/*μ*L)	1 *μ*l
10 mM dNTP mix	2 *μ*l
RevertAid RT (200 U/*μ*L)	1 *μ*l
Water, nuclease-free	9 *μ*l
Total volume	20 *μ*l

**Table 4:** The following table is showing the sequences of the chosen primer.

	Product	Primers	Tm (°C)	MW (g/Mol)	GC content
RAT	RAGE/F	AACCGGTGATGAAGGACAAG	57	6224	50
	RAGE/R	ATTCAGCTCTGCACGTTCCT	57	6018	50
	NFƙB/F	CGTCTGAAACTCTGGGAAGC	59	6142	55
	NFƙB/R	CCTCGCTGTTTAGGCTGTTC	59	6065	55
	IFN-*γ*/F	AGGAAAGAGCCTCCTCTTGG	59	6142	55
	IFN-*γ*/R	GGATCTGTGGGTTGTTCACC	59	6155	55
	TNF-*α*/F	ATGTGGAACTGGCAGAGGAG	59	6271	55
	TNF-*α*/R	GATCCTGGAGGGGAAGAGAC	60	6256	60
	GAPDH/F	ACAGCAACAGGGTGGTGGAC	60	6216	60
	GAPDH/R	TTTGAGGGTGCAGCGAACTT	57	6188	50

MICE	RAGE/F	GAAGGCTCTGTGGGTGAGTC	61	6229	60
	RAGE/R	ATTCAGCTCTGCAGTTCTCT	55	6033	45
	NFƙB/F	TGAGCGTAGGTGATGAGTGC	59	6253	55
	NFƙB/R	CTGGTCCCGTGAAATACACC	59	6061	55
	IFN-*γ*/F	ACTGGCAAAAGGATGGTGAC	57	6215	50
	IFN-*γ*/R	GACCTGTGGGTTGTTGACCT	59	6155	55
	TNF-*α*/F	AAGATGGAGGAAGGGCAGTT	57	6295	50
	TNF-*α*/R	GACCTGTGGGTTGTTGACCT	59	6155	55
	GAPDH/F	GGGTCCCAGCTTAGGTTCAT	59	6124	55
	GAPDH/R	CATTCTCGGCCTTGACTGTG	59	6074	55

Human	RAGE/F	AGGGAAAGAGGGAGTCAAGC	59	6289	55
	RAGE/R	GTGGATTTGAGGAGAGGG	55	5699	55
	NFƙB/F	CTGGGCCTCTGTACTTTGGA	59	6115	55
	NFƙB/R	GCAGAGCTCAGCCTCATAGA	59	6111	55
	IFN-*γ*/F	TGCAGAGCCAAATTGTCT	51	5498	44
	IFN-*γ*/R	TGCTTTGCGTTGGACATT	51	5511	44
	TNF-*α*/F	ATGTGGCAAGAGATGGGG	55	5668	55
	TNF-*α*/R	CTCACACACATCTGTCT	50	5065	47
	GAPDH/F	ACCCAGAAGACTGTGGAT	53	5532	50
	GAPDH/R	TTTTAGACGGCAGGTCAG	53	5554	50

**Table 5:** The decrease in the ROS content at varying concentrations of nanoassemblies.

Sample	RFU VALUE	% decrease in ROS
Native BSA-MG-AGEs	2104.36 ± 1589	—
25 mM BSA-MG-AGEs	4302.68 ± 2002	51.0
AGEs+PFT-HSA-TFT-Cy7 (1 *μ*M)	3217.03 ± 1552	25.11
AGEs+PFT-HSA-TFT-Cy7 (3 *μ*M)	3033.9 ± 1003	29.49
AGEs+PFT-HSA-TFT-Cy7 (5 *μ*M)	2600.91 ± 1662	39.56
AGEs+PFT-Hcy-HSA-Cy7 (1 *μ*M)	3192.46 ± 1718	25.8
AGEs+PFT-Hcy-HSA-Cy7 (3 *μ*M)	2708.56 ± 1078	37.05
AGEs+PFT-Hcy-HSA-Cy7 (5 *μ*M)	2147.61 ± 960	50.09

## Data Availability

The data used to support the findings of this study are included within the article.

## Abbreviations

AGE: Advanced glycation end products
CML: Carboxymethylysine
2,4 DNPH: 2,4-dinitrophenylhydrazine
FBG: Fasting blood glucose
RAGE: Receptor for advanced glycation end product
PFT: Perfluorotoluene
TFT: Trifluorotoluene
ROS: Reactive oxygen species.
